# lncRNA-SNHG14 Promotes Atherosclerosis by Regulating ROR*α* Expression through Sponge miR-19a-3p

This article has been retracted.

**DOI:** 10.1155/2020/3128053

**Published:** 2020-08-25

**Authors:** Baoliang Zhu, Jing Liu, Ying Zhao, Jing Yan

**Affiliations:** ^1^Department of Physiology, Jining Medical College, Jining, Shandong, China; ^2^Department of Pharmacy, Jining Medical College, Jining, Shandong, China; ^3^Department of Biochemistry, Jining Medical College, Jining, Shandong, China

## Abstract

Coronary heart disease (CHD) is the most common cardiovascular disease with high prevalence, disability, and mortality. The balance between proliferation and apoptosis of vascular smooth muscle cells (VSMCs) plays a key role in the initiation of atherosclerosis. In this study, we found a significant decrease in the expression of lncRNA-SNHG14 in atherosclerotic plaque tissues of ApoE-/- mice. Overexpression of lncRNA-SNHG14 can inhibit VSMC proliferation while promoting apoptosis. There is a potential reciprocal regulatory relationship between lncRNASNHG14 and miR-19a-3p, which inhibit each other's expression in vascular smooth muscle cells. In addition, the luciferase reporter gene analysis results showed that there was a direct interaction between miR-19a-3p and the 3′UTR of ROR*α*. The results of qRT-PCR showed that the level of ROR*α* mRNA was significantly increased in the aortas treated with miR-19a-3p and SNHG14 compared with that treated with miR-19a-3p alone. In conclusion, we demonstrated that lncRNA-SNHG14 regulates the apoptosis/proliferation balance of VSMCs in atherosclerosis.

## 1. Introduction

Coronary atherosclerotic heart disease (CHD), referred to as coronary heart disease, is mainly due to the occurrence of atherosclerosis in the coronary artery, which makes the lumen narrow or obstructed [1, 2]. This heart disease is associated with coronary spasm, leading to myocardial ischemia, hypoxia, or necrosis [3]. CHD is the most common cardiovascular disease, which has become the number one killer of human health in the 21st century due to its high morbidity, high disability, as well as high mortality [4]. With the acceleration of the aging social process in China, the incidence of this disease has been increasing year by year. The latest data of WHO in 2017 show that as many as 17.7 million people succumb to cardiovascular disease (CVD) every year, making up about 30% of the total global deaths, among which CHD ranks first [5]. However, the causes and mechanisms of CHD are not completely clear, and there are still many shortcomings in the prevention and treatment of this disease, which cannot fundamentally curb the increasing trend of the incidence and mortality of CHD. In order to explore its pathogenesis, it is of great significance to carry out experimental studies, especially intervention studies on animal models.

Pathological changes of atherosclerosis (AS) are characterized by lipid deposition in the intima and subintima of large and middle arteries [6]. In addition, smooth muscle cell (SMC) migration to the intima, proliferation and matrix proliferation, and inflammatory cell infiltration are also involved. These processes lead to intimal thickening and the formation of atherosclerotic lesions or fibrolipid plaque lesions [7, 8]. The research and debate on the mechanism of AS has lasted for more than 160 years, forming a variety of theories and factions, such as lipid infiltration theory, injury-response theory, inflammatory response theory, macrophage receptor deletion theory, SMC-causing mutation theory, platelet aggregation, and thrombosis theory [9]. However, neither doctrine alone can comprehensively explain the occurrence nor development of AS. Vascular smooth muscle cells (VSMC) is an important cellular component of the vascular wall. During development and maturation, VSMC is responsible for vasoconstriction and relaxation and responds to the stimulation of hemodynamic and environmental signals to regulate blood pressure and control vascular homeostasis in the body [10–12]. VSMC has strong plasticity. Normal VSMCs have no significant activity of proliferation, migration, and secretion of extracellular matrix, which is called contractile/differentiated VSMCs. However, VSMCs exhibit significant proliferative and migratory activities when they are immature, when physiological conditions change (such as long-term exercise, pregnancy), or when they are under pathological conditions (such as hypertension), and synthesize a large amount of extracellular matrix, which is called secretory/proliferative VSMC at this time [13–15]. The proliferation and differentiation of VSMC is a key regulatory process that affects the maturation and development of the vascular system. When vascular intima is damaged, VSMC overproliferation, migration, and synthesis of a large number of cellular matrix can induce cardiovascular diseases such as vascular restenosis, hypertension, and atherosclerosis [16, 17].

Long noncoding RNAs (lncRNAs) refer to bioactive RNAs with a length of >200 bases that cannot be translated into proteins and display mRNA-like features such as 5′capping, splicing, and polyadenylation. Several studies have confirmed that lncRNAs become powerful bioregulators by regulating a series of cellular processes in the nucleus or cytoplasm [18, 19]. Recent evidence has emerged that a variety of lncRNAs are involved in the regulation of AS and inflammatory response. For example, Wu's team [20] found that the expression of lincRNA-p21 was downregulated in the ApoE knockout mouse AS model. By interfering with the gene expression in vitro, it was confirmed that lincRNA-p21 inhibited the proliferation of VSMC and monocyte macrophages and induced apoptosis. Hu et al. [21] found that RP5-833A20.1 is an lncRNA regulating the NFIA gene, which may reduce the expression of NFIA by inducing the expression of mi-38R2-5p. Overexpression of NFIA increased HDL, decreased LDL and VLDL, increased reverse transport of CHOL, and inhibited AS formation.

Recent studies have shown that lncRNA-SNHG14 is upregulated in gliomas participates in tumor proliferation and migration as an oncogene [22]. The expression of miR-19a-3p was downregulated in gastric cancer, acting as a tumor suppressor by regulating the expression of different genes [23]. Recent studies have shown that lncRNA-SNHG14 promotes microglial activation in cerebral infarction by regulating miR145-5p/PLA2G4a [24]. However, the expression of lncRNA-SNHG14 in atherosclerosis remains unclear, and the relationship between the two and the clinicopathological features of patients have not yet been published. Herein, we aimed at further revealing the role of lncRNA in cardiovascular diseases and its possible molecular mechanism by studying the role of lncRNA-SNHG14 in the pathological process of atherosclerosis.

## 2. Methods

### 2.1. Bioinformatics Analysis

The prediction module of the DIANA LncBase2 tool (https://omictools.com/diana-lncbase-tool) was used to predict lncRNA-SNHG14-miR-19a-3p interaction. Target relationships between miR-19a-3p and ROR*α* were predicted using miRanda and target Scan.

### 2.2. Mouse Studies

Clean C57BL/6J mice were purchased from Jining Medical College Laboratory Animal Center, and ApoE knockout (ApoE-/-) mice were purchased from Jining Medical College Laboratory Animal Center. The mice were raised in the SPF grade mouse feeding room of Jining Medical College Laboratory Animal Center. Animal husbandry meets relevant management requirements, and all animal operations meet the ethical requirements of laboratory animals. Genotypes were homozygous ApoE knockout mice detected by RT-PCR using the genomic DNA of rat tail tissue as a template. Then, 10 male suckling mice were fed in two cages after the end of lactation and fed with 60% high-fat diet for one month to induce atherosclerosis. This study was approved by the Ethics Committee on Animal Experiments of XX Hospital.

### 2.3. Cell Culture and Transfection

Human primary aortic smooth muscle cells (HA-VSMC) are adherent cells with large cell morphology, spindle shape, and slow growth. In order to make it grow better, SmGM smooth muscle cell growth medium consisting of smooth muscle cell basal medium (Lonza, USA) was used in this study. TM-2 Bullet Kit™ Cell culture medium and kit, the mixed cell culture medium was prepared according to requirements. After adding various growth factors, fetal bovine serum was added to make the serum concentration reach 5%, and finally, penicillin streptomycin was added to prevent cell contamination. RAW264.7 mouse macrophages were also adherent growth cells with small cell morphology and polygonal or round shape, which were routinely cultured in DMEM medium containing 8% fetal bovine serum. The cells were placed in an incubator with 5% CO_2_ at 37°C. After the cells grew to logarithmic phase, experiments were carried out.

To induce overexpression of lncRNASNHG14 in VSMCs, pcDNA3.1-lncRNA-SNHG14 vectors were transfected into the cells. To enhance the miR-19a-3p level, miR-19a-3p mimics were transfected. siRNA of lncRNA-SNHG14 and miR-19a-3p was used to knockdown the expression of lncRNASNHG14 and miR-19a-3p in VSMCs. The pcDNA3.1 empty vectors and scramble control sequences were used as negative transfection controls. One day before transfection, HA-VSMC/RAW264.7 cells were passaged and seeded on cell culture plates at a certain density. Ensure that the cells can grow to 75%-85% fusion within 24 hours, ready for transfection. Add 100 nM siRNA to 100 ml of Opti-MEM and mix gently. Mix the Lipofectamine reagent with 100 uL serum-free DMEM or Opti-MEM, dilute the 4 uL Lipofectamine RNAiMAX reagent, mix gently, and stand for 5 minutes at room temperature. The diluted siRNA and reagents were mixed and left for 20 minutes, and then the complex was added to the cell plate for subsequent experiments. If the cell line is sensitive, remove the complex and replace the medium after incubation for 4-6 hours to prevent cell death.

Both small interference sequence of specific targeting SNHG14 (named si-SNHG14) and negative control sequence (named si-NC) were designed and synthesized by Shanghai Gma Biotechnology Co., LTD. The specific sequences were si-SNHG14, forward: 5′-GCUGAUAUUUAAGGCACUATT-3′ and reverse 5′-UAGUGCCUUAAAUAUCAGCTT-3′. Si-NC forward: 5′-UUCUCCGAACGUGUCACGUTT-3′ and reverse 5′-AACGUGACACGUUCGGAGAATT-3′.

### 2.4. CCK-8 Assay

CCK-8 solution (CCK-8; Dojindo) was added to each well with 10 microliters. A cell-free pore with the appropriate amount of cell culture medium was set up; drugs and CCK-8 solution were as a blank control. HA-VSMC (1.5 h) and RAW264.7 (1 h) were incubated in the cell incubator and absorbance was measured at 450 nm.

### 2.5. Flow Cytometry Assay for Apoptosis

The cells were collected and stained with cimin V-FITC and propidium iodide after transfection for 48 h. With Guava_easyCyte flow cytometry instrument testing process cells apoptosis rate, built-in software was used for analysis.

### 2.6. Real-Time Quantitative PCR (qRT-PCR)

Total RNA was extracted from cells by TRIzol™ reagent. In order to detect the mRNA levels of lncRNA-SNHG14 and miR-19a-3p, reverse transcription PCR was carried out with the PrimeScript RT Master Mix kit. Next, SYBR premix EX Taq II was used to amplify and quantify the cDNA according to 2 microliters of 5 ∗ RT Buffer, 0.5 microliters Enzyme mix, 0.5 microliters Primer mix, 2 microliters RNA, 5 uL Rnase free water. Then, set the Takara reverse transcription instrument at 37°C for 5 min, 95°C for 5 min, 4°C for reverse transcription PCR. The qRT-PCR instrument runs the PCR program: preheating at 95°C for 2 min, 8 cycles at 95°C for 30 s, 60°C for 4 s, and 72°C for 30 s, followed by 40 cycles at 95°C for 30 s, 56°C for 45 s, 72°C for 30 s, heating, and unlinking the chain to detect the fluorescence intensity. The sequence of lncRNA-SNHG14 is lncRNA-SNHG14 F: 5′-GGGTGTTTACGTAGACCAGAACC-3′, R: 5′- CTTCCAAAAGCCTTCTGCCTTAG-3′. The primer sequences of GAPDH are F: 5′- CCAAAATCAGATGGGGCAATGCTGG-3′, R: 5′- TGATGGCATGGACTGTGGTCATTCA-3′; the primer sequences of miR-19a-3p are F: 5′- CGCTGTGCAAATCTATGCAA-3′, R: 5′-CGGCCCAGTGTTCAGACTAC-3′. The ROR*α* primer sequences are F: 5′-GCTTCGGCAGCACATATACTAAAAT-3′, R: 5′-CGCTTCACGAATTTGCGTGTCAT-3′.

### 2.7. Western Blot

The VSMC was cleaved with a RIPA buffer, and the total protein was collected. The protein was isolated by SDS-PAGE and transferred to the NC membrane using a conventional protocol. The membrane was sealed with 5% skim milk at room temperature for 2 hours and incubated with ROR*α* (ab60134, Abcam, 1 : 1000) and *β*-actin (ab8226, Abcam, 1 : 1000) primary antibody at 4°C for 12 hours. Wash the membrane and incubate it with HRP secondary antibody for 2 h at room temperature. The blotting was visualized using an electrochemical luminescent Western blot kit. The strip strength was quantified using ImageJ software.

### 2.8. Dual-Luciferase Reporter Assay

Add 70 microliter PLB (Obio Technology) into the hole to be tested, shake, and lyse for 15 min in the dark. Then, add 100 microliter LARI and 20 microliter cell lysate into the white 96-well plate together, and measure the fluorescence value of firefly after mixing. Later, add 100 uL Stop&Glo into the sample immediately, the fluorescence value measured again after mixing was the internal reference kidney fluorescence value. Finally, the intensity of fluorescence was expressed by the ratio of the firefly fluorescence value to the kidney fluorescence value.

### 2.9. Statistical Analysis

All data were expressed as mean standard deviation (mean SD). Unpaired Student *t*-test was used when comparing two groups of data, and one-way ANOVA was used to compare more than two groups of data. Statistical differences were considered when *P* < 0.05. Data statistics and plotting were performed using SPSS17.0 and GraphPad Prism 5.0.

## 3. Results

### 3.1. Expression of lncRNA-SNHG14 in Atherosclerotic Plaques

Atherosclerosis was successfully induced in ApoE-/- mice fed a 60% high-fat diet for one month. Total RNA from atherosclerotic plaque tissues of male ApoE-/- mice and aortic vascular tissues of normal C57BL/6J mice was extracted and quantified by qPCR. We found that compared with wild-type C57BL/6J mice, the expression of lncRNA-SNHG14 in atherosclerotic plaque tissue of ApoE-/- mice was significantly reduced, as shown in Figure 1(a). After transfection of siRNA against murine and human lncRNA-SNHG14 in RAW264.7 cells and HA-VSMC cells, respectively, the expression of lncRNA-SNHG14 was successfully knocked down in both cells by qPCR detection, as shown in Figure 1(b).

### 3.2. Detection of the Role of lncRNA-SNHG14 in Cell Proliferation and Apoptosis

To further clarify the function of lncRNA-SNHG14, we transfected siRNA against murine and human lncRNA-SNHG14 in RAW264.7 cells and HA-VSMC cells. After cell counting detection, we found that the number of both cells increased significantly 48 hours after transfection compared with the siRNA transfection group with unrelated sequence after lncRNA-SNHG14 silencing (Figure 2(a)). After the transfection of siRNA targeting murine and human lncRNA-SNHG14 in RAW264.7 cells and HA-VSMC cells, CCK-8 cell proliferation assay indicated that the proliferation level of the two cells was significantly increased 48 hours after transfection compared with the siRNA control group after lncRNA-SNHG14 silencing (Figure 2(b)).

In addition, we also transfected siRNA against murine and human lncRNA-SNHG14 in RAW264.7 cells and HA-VSMC cells, respectively, and detected apoptosis by flow cytometry. We found that after lncRNA-SNHG14 silencing, the apoptotic level of the two cells was significantly lower than that of the siRNA control group, indicating that the silencing of lncRNA-SNHG14 inhibited the apoptosis of the two cells (Figure 2(c)).

### 3.3. Interaction between lncRNA-SNHG14 and miR-19a-3p

To verify whether there is a regulatory relationship between lncRNA-SNHG14 and miR-19a-3p, we performed targeted binding prediction between LncRNA SNHG14 and miR-19a-3p (Figure 3(a)). In addition, we transfected lncRNA-SNHG14 overexpression plasmid or infected with miR-19a-3p lentivirus on vascular smooth muscle cells. The results showed that the upregulation of lncRNA-SNHG14 could significantly inhibit the expression of miR-19a-3p. When the expression of miR-19a-3p was upregulated, the expression of lncRNA-SNHG14 was also inhibited. This suggests that lncRNA-SNHG14 and miR-19a-3p inhibit each other's expression in vascular smooth muscle cells, and there is a potential mutual regulatory relationship between the two (Figure 3(b)).

We constructed dual-luciferase reporter plasmids containing the sequences of wild-type and mutant (in which all three potential binding targets were mutated) of the potential targeting binding sites of miR-19a-3p and lncRNA-SNHG14 to verify their binding in vivo. Luciferase assay found that the relative fluorescence activity of wild-type luciferase plasmid decreased significantly compared to the mutant group (Figure 3(c)). Subsequently, we validated the binding in vitro of lncRNA-SNHG14 to miR-19a-3p by RNA pull-down assay. It was found that the biotin-labeled lncRNA-SNHG14 sense strand could pull out more miR-19a-3p than lncRNA-SNHG14 antisense strand. The binding and adsorption of lncRNA-SNHG14 on miR-19a-3p were further illustrated (Figure 3(d)).

### 3.4. SNHG14/miR-19a-3p Promotes VSMC Proliferation and Inhibits Its Apoptosis by Targeting ROR*α*

Through bioinformatics prediction analysis, there is a binding site of miR-19a-3p in the 3′UTR of ROR*α*, and it is speculated that ROR*α* may be a downstream target of SNHG14 to play a regulatory role through miR-19a-3p (Figure 4(a)). The results of luciferase reporter gene analysis showed that there was a direct interaction between miR-19a-3p and the 3′UTR of ROR*α* (Figure 4(b)). Furthermore, Western Blot assay showed that after overexpression of miR-19a-3p, the expression of ROR*α* decreased compared with the control group (*P* < 0.05), confirming that ROR*α* can be used as a regulatory target of miR-19a-3p (Figure 4(c)).

We injected the SNHG14 overexpression plasmid with adenovirus pMIR-19a-3p and the corresponding control tail vein into ApoE-/- mice and aortic tissues, respectively. The results of qRT-PCR showed that the level of ROR*α* mRNA was significantly increased in the aortas treated with miR-19a-3p and SNHG14 compared with that treated with miR-19a-3p alone (Figure 5(a)). Western blot also showed that the expression of ROR*α* protein in the aorta treated with SNHG14 and miR-19a-3p was higher than that in the tissues treated with only miR-19a-3p, but lower than that in the tissues treated with only SNHG14. The result suggests that SNHG14 can reverse the inhibitory effect of miR-19a-3p on the expression of ROR*α* in the liver and aorta of ApoE -/- mice (Figure 5(b)).

## 4. Discussion

LncRNA-SNHG14, also known as UBE3A-ATS, is located on human chromosome 15q11.2. Knockout of the SNHG14 gene significantly inhibits the survival, migration, invasion, and promotes apoptosis of gastric cancer SGC-7901 cells [25]. Studies in renal cancer have found that lncRNA-SNHG14 is upregulated and can be used as a ceRNA to promote the migration and invasion of clear cell renal cancer [26]. Qi and other studies have shown that lncRNA-SNHG14 promotes microglial activation by regulating miR145-5P/PLA2G4a and participates in the occurrence of cerebral infarction [24]. The study confirmed that the expression level of lncRNA-SNHG14 in the serum of acute cerebral infarction was upregulated, and with the aggravation of acute cerebral infarction, the expression level of lncRNA-SNHG14 gradually increased, suggesting that lncRNA-SNHG14 participates in the occurrence and progression of acute cerebral infarction. However, to our knowledge, there is no published evidence that lncRNA-SNHG14 is associated with dysfunction of VSMC in atherosclerosis. We examined the expression of lncRNA-SNHG14 in patients and analyzed its function in vitro. As expected, downregulated lncRNA-SNHG14 was observed in the AS mouse model, and lncRNA-SNHG14 could inhibit VSMC proliferation but induce apoptosis. These results suggest that lncRNA-SNHG14 plays a role in atherosclerosis and may be used as a potential target for therapy. The mechanism by which lncRNA-SNHG14 regulates proliferation/apoptosis deserves further study. However, the molecular functions performed by lncRNAs and the corresponding mechanisms are essentially complex. To simplify the problem, we only tried a popular theory called ceRNA theory to partially explain how lncRNA-SNHG14 performs its function. In brief, we established a model of lncRNA-microRNA-mRNA regulation based on the concept of ceRNA, and designed experiments to confirm whether certain mechanisms are suitable for this model. In addition, we performed a bioinformatics analysis to understand the potential interaction between lncRNA-SNHG14 and microRNA. Using the DIANA LncBase2 tool, we speculated that >200 microRNAs might interact with lncRNA-SNHG14.Among these candidate microRNAs, we chose miR-19a because it is fully studied in the regulation of VSMC function.

miRNAs are a class of endogenous noncoding small RNAs with a length of 21-25 nucleotides, which can cleave or repress target gene mRNAs by binding to the 3′-non-coding region of target mRNAs.MiR-19a is located in chromosome region 13q31.3 and has been confirmed to be associated with malignant transformation of metastatic breast and colon cancer [27, 28]. Studies have shown that in hyperlipidemia, mildly oxidized LDL can stimulate HIF-1a expression in vascular endothelial cells, and endothelial HIF-1a can trigger miR-19a-mediated CXCL1 expression and monocyte adhesion to promote atherosclerosis progression [29]. miR-19a is an important member of the polycistronic gene cluster of miR-17-92. Current studies have found that the gene cluster in which miR-19a resides can be activated during atherosclerosis, promoting vascular inflammation and foam cell formation [30]. miR-19a was also found to be upregulated in endothelial vascular cells under hypoxia-inducible factors and shear stress, increasing the proliferation and antiapoptotic ability of endothelial vascular cells [29]. Animal models of atherosclerosis provide more evidence for the role of miR-19a in vivo. ApoE-/- mice fed a high-fat diet were treated with an antagonist of miR-19a, which is consistent with our findings. Histological analysis of thoracic and abdominal aorta specimens revealed that atherosclerotic plaques and lipid content were significantly reduced in mice [31]. The above evidence suggests that inhibition of miR-19a can alleviate the inflammatory response and slow down the development of atherosclerosis. At present, it has been reported that miR-19a is elevated in serum and atherosclerotic lesions of patients with coronary artery disease, which may be one of the initiating factors of atherosclerosis [32].

Nuclear receptors are a class of ligand-dependent transcription factor superfamily. Retinoic acid-related orphan receptors (RORs) are named for their similarity in gene sequence to retinoic acid receptors (RARs) and retinoid X receptors (RXRs). RORs include three subfamilies: ROR*α*, ROR*β*, and ROR*γ*. Because the endogenous ligands of RORs receptors are unknown, they are called orphan nuclear receptors. Through the study of ROR*α* molecular structure, action characteristics, and ROR*α* gene mutation deficient (ROR*α*sg/sg) mice, we found that ROR*α* plays an important role in the regulation of lipid metabolism. Compared with wild-type mice, the serum triglyceride (TG), total cholesterol (TC), and high-density lipoprotein (HDL) of ROR*α* sg/sg mice were lower under normal dietary conditions [33, 34], which indicated that ROR*α* was closely related to lipid metabolism. Abnormal expression of ROR*α* can cause metabolic disorders, leading to an increased prevalence of various metabolic-related diseases, including obesity, type 2 diabetes, atherosclerosis, and so on. When atherosclerosis occurs, ROR*α* expression is significantly reduced in smooth muscle cells and endothelial cells. Vascular smooth muscle cell apoptosis and extracellular matrix homeostasis are key links in regulating atherosclerotic plaque stability. When unstable plaques are formed, the phagocytic clearance of apoptotic cells by macrophages is defective or inadequate, leading to decreased clearance of apoptotic cells. The increase of apoptotic cells and the decrease of macrophage's funeral effect on apoptotic cells make a large accumulation of apoptotic cells in plaque, which will promote the further release of inflammatory factors and matrix-degrading enzymes, trigger the expansion of necrotic core, further thinning and rupture of plaque fibrous cap, and promote the occurrence of acute coronary events.

In this study, we first used ApoE knockout mice to detect the expression of SNHG14 in atherosclerotic plaques by qRT-PCR after atherosclerosis was induced by high-fat diet feeding. We found that the expression of SNHG14 in atherosclerotic plaque tissues of ApoE-/- mice was significantly decreased compared with wild-type C57BL/6J mice. Thus, the possible correlation between SNHG14 and AS was preliminarily verified. Next, we used mouse macrophage cell line RAW264.7 and human primary cultured aortic vascular smooth muscle cell HA-VSMC. The cell model of SNHG14 gene silencing was prepared by siRNA transfection, and then the levels of cell proliferation and apoptosis were detected in vitro. Results after silencing SNHG14 in RAW264.7 cells and HA-VSMC cells, the proliferation level of the above two cells increased while the apoptotic level was inhibited. This finding indicates that SNHG14 can affect the proliferation and apoptosis of the above two AS-related cells at the in vitro level. In addition, the upregulation of lncRNA-SNHG14 can cause changes in the microRNA 19a-3p/ROR*α* axis. Combined with the results of bioinformatics analysis and dual-luciferase reporter gene experiment, we believe that lncRNA-SNHG14 has the potential of sponge adsorption of microRNA-19a-3p.

It has been reported that both microRNA-19a-3p and ROR*α* are involved in regulating the function of VSMCs in atherosclerosis, thus indirectly confirming the possible target relationship between microRNA-19a-3p and ROR*α*. These results suggest that there may be a regulatory mode of lncRNA-SNHG14/microRNA-19a-3p/ROR*α* in the dysfunction of atherosclerotic VSMCs.

## 5. Conclusion

In conclusion, we believe that lncRNA-SNHG14 is an important regulator of vascular smooth muscle cell proliferation and apoptosis in the process of atherosclerosis. lncRNA-SNHG14 can exert this function by regulating the microRNA-19a-3p/ROR*α* axis as ceRNA. Restoring the expression of lncRNA-SNHG14 in vascular smooth muscle cells may be a potential target for atherosclerotic treatment.

## Figures and Tables

**Figure 1:** Expression of lncRNA-SNHG14 in atherosclerotic plaques. (a) Expression of lncRNA-SNHG14 in mouse atherosclerotic plaques. WT: 5 normal C57BL/6 mice; ApoE-/-: 5 ApoE-/- knockout mice, ^∗^*P* < 0.05. (b) Detection of lncRNA-SNHG14 expression in RAW264.7/HA-VSMC cells. Cntl-siRNA was the irrelevant sequence siRNA control transfection group, si-mlncRNA-SNHG14 was the siRNA transfection group for mouse lncRNA-SNHG14, si-hlncRNA-SNHG14 was the siRNA transfection group for human lncRNA-SNHG14, ^∗^*P* < 0.05.

**Figure 2:** Detection of the role of lncRNA-SNHG14 in cell proliferation and apoptosis. (a) Cell counts of RAW264.7/HA-VSMC cells at different time points after lncRNA-SNHG14 silencing. Left: RAW264.7 cells; Right: HA-VSMC cells. The ordinate represents the relative cell number; the harvesting time of 0, 24, 48, 72 cells after transfection, in hours. (Cntl-siRNA was the irrelevant sequence siRNA control transfection group, si-mlncRNA-SNHG14 was the siRNA transfection group for mouse lncRNA-SNHG14, si-hlncRNA-SNHG14 was the siRNA transfection group for human lncRNA-SNHG14, ^∗^*P* < 0.05). (b) Cell proliferation detection of RAW264.7/HA-VSMC cells at different time points after lncRNA-SNHG14 silencing. Left: RAW264.7 cells; Right: HA-VSMC cells. The ordinate represents the relative absorbance value; the harvesting time of 0, 24, 48, 72 cells after transfection, in hours. (Ctl-siRNA was the irrelevant sequence siRNA control transfection group, si-mlncRNA-SNHG14 was the siRNA transfection group for mouse lncRNA-SNHG14, si-hlncRNA-SNHG14 was the siRNA transfection group for human lncRNA-SNHG14, ^∗^*P* < 0.05. (c) Detection of apoptosis in RAW264.7/HA-VSMC cells after lncRNA-SNHG14 silencing. Flow cytometry two-dimensional dot plot and Flow cytometry two-dimensional dot plot data statistical graph. The ordinate of the two-dimensional dot plot of flow cytometry data is the percentage of apoptotic cells. Cntl-siRNA was an irrelevant sequence siRNA control transfection group, and si-lncRNA-SNHG14 was a siRNA transfection group for mouse or human lncRNA-SNHG14, ^∗^*P* < 0.05.

**Figure 3:** Interaction between lncRNA-SNHG14 and miR-19a-3p. (a) Targeted binding between LncRNA SNHG14 and miR-19a-3p. (b). Left: the expression result of miR-19a-3p when overexpressing LncRNASNHG14; Right: the expression result of lncRNASNHG14 when overexpressing miR-19a-3p; ^∗^*P* < 0.05, ^∗∗^*P* < 001. (c) Analysis results of fluorescence data after cotransfection of mimic with dual luciferase plasmid; (d) RNA pull-down validates the binding of miR-19a-3p to lncRNA SNHG14; ^∗^*P* < 0.05, ^∗∗^*P* < 0.01.

**Figure 4:** SNHG14/miR-19a-3p promotes VSMC proliferation and inhibits its apoptosis by targeting ROR*α*. (a) Patterns of construction of wild-type and mutant dual-luciferase plasmids; the red part is the mutated base site; (b) Analysis results of fluorescence value data after cotransfection of mimic and dual-luciferase plasmids; ^∗∗^*P* < 0.1. (c) Relative expression of RORalpha protein in cells; ^∗^*P* < 0.05, ^∗∗^*P* < 0.01.

**Figure 5:** Overexpression of SNHG14 reverses the inhibition of RORalpha mRNA (a) and protein (b) levels in ApoE-/- mouse aorta by miR-19a-3p. Note: ^∗^*P* < 0.05 vs. miR-NC group; ^#^*P* < 0.05 vs. miR-19a-3p group.

## Data Availability

The related data can be provided if any researchers required.
